The article "Low Serum Vitamin D Is Associated with Anti-Thyroid-Globulin Antibody in Female Individuals" was published in 2015. Journal: Int J Endocrinol.

# Low Serum Vitamin D Is Associated with Anti-Thyroid-Globulin Antibody in Female Individuals

**DOI:** 10.1155/2015/285290

**Published:** 2015-11-22

**Authors:** Xinling Wang, Jazyra Zynat, Yanying Guo, Reziwan Osiman, Aihemaitjan Tuhuti, Hongli Zhao, Munira Abdunaimu, Huili Wang, Xiaoping Jin, Shuqing Xing

**Affiliations:** Department of Endocrinology, People's Hospital of Xinjiang Uyghur Autonomous Region, Urumqi 830000, China

## Abstract

*Objectives*. Some evidence has pointed out that vitamin D plays a significant role in reducing the incidence of autoimmune diseases, especially autoimmune thyroid diseases. The authors aimed to examine the relationship between circulating 25-hydroxyvitamin D and thyroid autoantibody in a population-based health survey of Xinjiang Chinese population.* Subjects and Methods*. A total of 1714 Chinese adults were analyzed. 25(OH)D, anti-thyroid antibodies, and thyroid function were measured.* Results*. The prevalence of vitamin D insufficiency was 28.3% in Hans and 9.3% in Uyghurs, and the prevalence of vitamin D deficiency was 61.6% in Hans and 87.6% in Uyghurs. Overall prevalence of TgAb positivity was 6.2% (0.9% males; 5.3% females). In female subjects, mean serum 25(OH)D levels were significantly lower in Hans and Uyghurs compared with males, and the difference was statistically significant. Importantly, after adjusting for age and ethnicity, a negative correlation (*r* = −0.121, *P* = 0.014) was recognized between 25(OH)D and TgAb levels only in female subjects.* Conclusion*. Vitamin D insufficiency and deficiency are prevalent among Chinese adults. Low serum 25(OH)D is related to the presence of TgAb in females. The causal effect of low vitamin D level on thyroid autoimmunity should be studied further more.

## 1. Introduction

Vitamin D insufficiency and/or deficiency are becoming a global health problem. Its role as an immune modulator has been recently emphasized. Many studies provide evidence pointing to a clear role of vitamin D in the pathogenesis of autoimmune diseases, especially autoimmune thyroid diseases (AITDs), as vitamin D deficiency is linked with high levels of anti-thyroid antibodies, abnormal thyroid function, increased thyroid volume, and increased TSH levels [1–4]. Nevertheless, at the present time vitamin D levels above 30 ng/mL are considered sufficient and confer protection from bone disease, whereas lower levels induce elevation of parathyroid hormone and are associated with other hazardous systemic effects [5]. However, it is unclear whether low vitamin D levels are closely associated with the development of autoimmune thyroid disease. Some case-control studies have suggested that lower serum vitamin D levels or a higher prevalence of vitamin D insufficiency existed in patients with AITDs compared with that in healthy controls [1, 2, 6, 7]. However, another study reported no significant association between serum vitamin D levels and thyroid autoimmunity [4]. Thus, we aim to estimate the associations between vitamin D deficiency and/or insufficiency and autoimmune thyroid diseases, especially to clarify the relationship between vitamin D and serum thyroid autoantibody, in a relative rather than quantitative manner by comparing levels of vitamin D in a Chinese population.

The article "Low Serum Vitamin D Is Associated with Anti-Thyroid-Globulin Antibody in Female Individuals" was published in 2015. Journal: Int J Endocrinol.

## 2. Subjects and Methods

### 2.1. Study Population

From May to June 2013 this study was performed in Ürümqi of Xinjiang province. Adults aged 16 years and above who were Chinese citizens and lived in current residence for 3 years or longer were selected and invited into our study. Those with severe communication problems and acute illness and unwilling to participate were excluded from the study. A total of 2253 people participated in this investigation (Figure 1). We excluded participants who had missing lab results (*n* = 140) and questionnaire data (*n* = 153) and were younger than 16 years old (*n* = 4) and other ethnic groups (*n* = 242). Finally, 1714 subjects were enrolled, including Han and Uyghur. The study protocol was approved by the Ethics Committee of People's Hospital of Xinjiang Uyghur Autonomous Region. Informed consent was obtained from all subjects before data collection.

In our study site, all the data collection was performed by the same staff group from Department of Endocrinology in People's Hospital of Xinjiang Uyghur Autonomous Region. They were trained according to a standard protocol that made them familiar with the specific tools and methods used. Venous blood samples were drawn after an overnight fast of at least 8 h and centrifuged on the spot after collection. Blood samples were collected and stored at −80°C.

### 2.2. Laboratory Tests

Serum 25(OH)D levels and thyroid parameters, serum TSH, and the levels of TgAb and TPOAb were measured with a Roche electrochemiluminometric analyzer (E601), with an interassay variance of <10%. It is generally agreed that serum 25(OH)D levels of 20 to 30 ng/mL should be considered as representative of vitamin D insufficiency, whereas serum 25(OH)D levels of <20 ng/mL should be considered as an indicative of vitamin D deficiency [8]. Serum TPOAb of >35 IU/mL and/or TgAb of >116 IU/mL were considered autoantibody positivity (Roche).

### 2.3. Statistical Analysis

Continuous variables are presented as means ± standard deviation for continuous normally distributed variables and median (interquartile range) for the nonnormally distributed variables. Student's *t*-test and Mann-Whitney *U* test were used for comparison of mean values between groups. Linear regression analysis was used to examine the relationship between log-transformed TgAb/TPOAb titer and age, ethnicity, 25(OH)D, and other biochemical variables. Multivariate regression analysis was performed to identify the predictive variables. All calculations were performed using SPSS 19.0 for Windows (Chicago, IL, USA). A probability (*P*) value of <0.05 was considered statistically significant for all tests.

The article "Low Serum Vitamin D Is Associated with Anti-Thyroid-Globulin Antibody in Female Individuals" was published in 2015. Journal: Int J Endocrinol.

## 3. Results

A total of 1,714 subjects (969 Han and 745 Uyghur) including 1,197 females (652 Han and 545 Uyghur) and 517 males (317 Han and 200 Uyghur) were enrolled in this study. The mean level of total serum 25(OH)D was 16.55 ± 8.53 ng/mL. Vitamin D deficiency and insufficiency were noted in 1250 (72.9%) and 344 (20.1%) subjects, respectively.

### 3.1. Clinical and Laboratory Characteristics

Females had higher serum TSH levels and TPOAb and TgAb titres but lower serum 25(OH)D levels than males (*P* < 0.05) (Table 1). Ethnic subgroup studies showed that Uyghurs had higher TPOAb and TgAb titres but lower serum TSH and 25(OH)D levels compared to Hans (*P* ≤ 0.001). Han subjects were significantly older than Uyghurs (48.34 ± 15.46 versus 43.78 ± 12.81 years, *P* < 0.01). Vitamin D insufficiency was noted in 28.3% of Han and 9.3% of Uyghur residents and vitamin D deficiency was seen in 61.6% of Hans versus 87.6% of Uyghurs. As shown in Figure 2, Uyghurs had a lower mean 25(OH)D level compared to Hans (19.40 ± 8.37 versus 12.84 ± 7.23, *P* < 0.001). In the ethnic Han subgroup, females had a lower mean 25(OH)D level compared to males (19.18 ± 8.88 versus 19.86 ± 7.18 ng/mL, *P* = 0.002); similarly Uyghur females had lower 25(OH)D levels than Uyghur males (11.67 ± 7.28 versus 16.04 ± 6.01 ng/mL, *P* < 0.001).

### 3.2. Clinical and Laboratory Characteristics of Positive Serum Thyroid Antibodies

In the present study, 240 (14.0%) subjects were positive for serum TPOAb and a total of 106 (6.2%) subjects were positive for serum TgAb, of which 209 (12.2%) were positive for both serum TPOAb and serum TgAb. There were a significant high proportion of females compared to males in TPO(+), Tg(+), and TPO(+)Tg(+) groups (73.3% versus 26.7%, *P* = 0.203; 85.8% versus 14.2%, *P* < 0.001; 86.6% versus 13.4%, *P* < 0.001; resp.), while the proportion of Uyghurs was higher as compared to Hans (*P* < 0.05) only in the Tg(+) group but not in the TPO(+) and TPO(+)Tg(+) groups. TgAb(+) group had a lower mean 25(OH)D level compared to the TgAb(−) group (*P* < 0.01). The prevalence of vitamin D deficiency in TgAb positive subjects was higher than that observed in TgAb negative subjects, while no statistical difference was found (78.3% versus 72.6%, *P* = 0.199). The serum TSH levels in the TPO(+)Tg(+) group were significantly higher than those in the TPO(+) group and Tg(+) group (*P* < 0.01). However, there was no significant difference between TPO(+) group and Tg(+) group (Table 2).

The article "Low Serum Vitamin D Is Associated with Anti-Thyroid-Globulin Antibody in Female Individuals" was published in 2015. Journal: Int J Endocrinol.

### 3.3. Relationship between Serum 25(OH)D Levels and Anti-Thyroid Antibodies

To account for the probable interaction between vitamin D status and anti-thyroid antibody level, further analyses were performed according to gender differences. It was found that higher TgAb titres were associated with lower 25(OH)D levels independent of age, ethnicity, and TSH levels in females (beta = −0.121, *P* = 0.014, Table 3) but not in males. Linear regression analysis showed a weak relationship between TPOAb titres and serum 25(OH)D levels independent of age, ethnicity, and TSH levels (males, beta = 0.005, *P* = 0.002; females, beta = 0.006, *P* = 0.000, Table 4). Age, TSH, and thyroid-globulin antibody titres, but not 25(OH)D or ethnicity, were associated with TPOAb titres in men and women.

Given the findings of lower serum 25(OH)D levels in female subjects in the TgAb(+) group, we evaluated the adjusted odds ratios (ORs) for women using multivariate logistic regression model. The multivariate analysis using logistic regression revealed that 25(OH)D levels were an independent determinant of the presence of TgAb (odds ratio: 1.156, 95% confidence interval: 1.004–1.331, *P* = 0.043; see Table 5) after adjusting for age, gender, and ethnicity. In this analysis, gender, ethnicity, and TSH showed a significant association with TgAb positivity. However, age had no significant association.

## 4. Discussion

In the current study, we found that a low circulating 25(OH)D level was significantly associated with a higher risk of prevalent AITDs in females. To the best of our knowledge, this is the first study to investigate the association between circulating 25(OH)D and anti-thyroid antibodies in community based men and women from Xinjiang province of China.

According to our study performed, the mean serum vitamin D level in the Xinjiang population is 16.55 ± 8.53 ng/mL, and the prevalence of vitamin D deficiency is 72.9%. This prevalence is remarkably high in the Uyghur population, especially in Uyghur females compared to males. Wearing covered clothing was reported to be associated with lower 25(OH)D levels [9]. The fact that vitamin D deficiency is predominantly found in Uyghur females signifies a certain association between these two conditions; it seems that the lower 25(OH)D level in Uyghurs is due to headscarves and clothing that covers the neck, arms, and legs. In contrast, Han populations are more mindful of their health and often exercise outdoors before and after work and with ordinary clothing, thereby increasing their sunshine exposure.

The article "Low Serum Vitamin D Is Associated with Anti-Thyroid-Globulin Antibody in Female Individuals" was published in 2015. Journal: Int J Endocrinol.

Lower vitamin D levels have been found in several autoimmune diseases, such as rheumatoid arthritis, systemic lupus erythematosus, systemic sclerosis, type 1 diabetes mellitus, multiple sclerosis, inflammatory bowel diseases, autoimmune thyroid diseases (i.e., Hashimoto's thyroiditis and Graves' disease), and autoimmune gastritis [10]. The mechanisms underlying the link between vitD and autoimmunity are not completely understood but probably are associated with its anti-inflammatory and immunomodulatory functions, as well as the presence of VDRs on most immune cells [10, 11]. AITDs are multifactorial diseases in which autoimmunity plays a fundamental role with infiltration of the gland by T- and B-cells and production of specific autoantibodies, reactive to thyroid antigens [antithyroglobulin, anti-thyroid peroxidase (TPOAb), and anti-TSH receptor (TRAb)] [12]. Kivity et al. [1] reported, for the first time, a link between vitamin D deficiency and the presence of anti-thyroid antibodies. In recent years, evidence has emerged pointing to an involvement of vitamin D in the development of autoimmune thyroid disease [13]. The immune modulator properties of vitamin D are ascribed to its effect on cells of the innate and adaptive systems, including macrophages, dendritic cells, and T and B lymphocytes, all of which harbor VDR [11]. Recently, several genetic studies have demonstrated an association between thyroid autoimmunity susceptibility and gene polymorphisms of numerous proteins and enzymes that are associated with vitD functions, including VDR, DBP, CYP27B1, and CYP2R1 [11, 12, 14]. Activated vitamin D modulates autoimmune reactions by regulating T lymphocytes to inhibit both the production and activity of cytokines [15]. Vitamin D directly regulates T lymphocyte functions by inhibiting the proliferation of Th1 cells and increasing the number of Th2 cells [16]. Vitamin D also suppresses the production of IL-2, IL-5, IFN-c, and TNF-a and increases the production of IL-4 and transforming growth factor in Th2 cells [17]. There are no further experimental studies to reveal whether there is a casual relationship and what are the mechanisms between low serum vitamin D and anti-thyroid antibody presence. Hence, from the results of our study, we supposed that vitamin D may enhance the responsiveness in thyroid autoimmune reaction which induced TgAb secretion of thyrocytes.

In the present study, the prevalence of vitamin D deficiency (78.3%) and insufficiency (20%) is higher in TgAb positive subjects. In addition, we explored the probable interaction between vitamin D status and thyroid-globulin antibodies in female Xinjiang Chinese population. Similar to the study in other populations, it has been observed that women have higher serum antithyroglobulin antibody (TgAb) levels but lower serum 25(OH)D levels than men [3]. It is reported that vitamin D deficiency is more closely related to anti-thyroid antibody titer rather than thyroid function itself in humans [18]. Our study not only supports the existing argument on the association between vitamin D and AITDs but also further solidifies the association by revealing that 25(OH)D has a statistical correlation with TgAb presence.

The article "Low Serum Vitamin D Is Associated with Anti-Thyroid-Globulin Antibody in Female Individuals" was published in 2015. Journal: Int J Endocrinol.

Our current results suggest a possible crosstalk between vitamin D and X chromosome in the development of AITDs. The association of lower vitamin D levels with the higher prevalence of TgAb positivity was found to be significant only in women and not in men, which is likely to more accurately reflect the mean reference value of serum 25(OH)D and the relationship with TgAb. AITDs have a female : male ratio of approximately 9 : 1 [19]. There is also some studies that provide strong evidence for female predominance and X chromosome involvement in AITDs, such as the finding that the X chromosome contains a considerable number of sex and immune-related genes that are essential in determining sex hormone levels and more importantly in immune tolerance, such as AR, IL-2 receptor gamma chain, CD40 ligand, and FOXP3 [20–22]. An alternative explanation has been recently proposed, that is, an enhanced skewed XCI in peripheral blood cells of female patients with autoimmune diseases [23–26]. Results from our study showed a significant high proportion of women in Tg(+) group, which is consistent with previous studies, making better understanding of AITDs occurrence risks from the perspective of sex determination genetics in females compared to males. The X chromosome has been a recurrently suspicious contributor to disease genetics, and many reports provide strong evidence that the prevalence of vitamin D deficiency or insufficiency was more severe in female individuals. Further clinical and experimental investigations of the effect of vitamin D supplementation on thyroid antibodies, particularly in female individuals, are needed to elucidate an effect of vitamin D on either the thyrocytes or the thyroid follicular epithelium and genetic differences that might provide insight into this relationship.

Most of the studies supported the inverse relation between low levels of 25(OH)D and autoimmune disease [10–12]. Interestingly, in our study multivariate logistic regression analysis revealed that 25(OH)D was an independent risk factor of TgAb. We suppose that this result of the study indicated that both low and high levels of vitamin D may result in an increased prevalence of autoimmune thyroid diseases. Some studies have investigated the association between mortality and higher levels of 25(OH)D and found both high and low levels of 25(OH)D were associated with increased risk of overall mortality [27, 28]. Durup et al. suggested a U-shaped relationship between serum 25(OH)D concentration and the frequency of certain pathologies [29]. Unfortunately, the appropriate range for vitamin D that will be safe and sufficient to modulate immunological homeostasis is yet to be determined.

The article "Low Serum Vitamin D Is Associated with Anti-Thyroid-Globulin Antibody in Female Individuals" was published in 2015. Journal: Int J Endocrinol.

It is generally agreed that high serum 25(OH)D levels are associated with low circulating TSH. Recently, population-based studies have reported that high vitamin D status in younger individuals and middle-aged and elderly males is associated with low circulating thyroid-stimulating hormone (TSH) [3, 30]. However, our study did not find a link between vitamin D status and thyrotropin after controlling for age, gender, ethnicity, and thyroid autoantibody. The lack of statistical significance may be due to the relatively small number of subjects, especially after subgroup analysis in different ethnics or genders.

Our study is limited by the fact that we did not record several factors affecting sun exposure, such as outdoor activity, difference in the use of sunscreens, and vacation activities. In our study, serum 25(OH)D was measured at the end of spring season in the Xinjiang region of China; the average amount of sunshine for May and June was up to 13-14 hours. However, our findings strongly suggest that we likely underestimate vitamin D deficiency in the population. Another limitation is the lack of information on differences in socioeconomic status between Hans and Uyghurs in this cohort. Besides, because of the cross-sectional nature of the present study, the causative effect of vitamin D on serum anti-thyroid-globulin antibody titres could not be readily determined.

## 5. Conclusion

Vitamin D insufficiency or deficiency is common among Chinese adults. 25(OH)D status was much worse among Uyghur (especially in females) populations, the prevalence of vitamin D deficiency and insufficiency was higher in TgAb positive individuals, and low serum 25(OH)D was associated with TgAb presence only in female subjects. Taken together, these data suggest a pathogenic relationship between vitamin D status and AITDs. Future studies are warranted to clarify the potential contribution of the low serum vitamin D to the development of autoimmune thyroid diseases.

The article "Low Serum Vitamin D Is Associated with Anti-Thyroid-Globulin Antibody in Female Individuals" was published in 2015. Journal: Int J Endocrinol.

## Figures and Tables

**Figure 1:** Flow diagram of participant enrollment in our study.

**Figure 2:** Serum levels of serum 25(OH)D in the study subjects according to the gender and ethnicity.

**Table 1:** Clinical characteristics for the participants.

	Ethnicity	Male	Female	*P* value
Age	Han	45.05 ± 17.47	49.99 ± 14.11	0.000
	Uyghur	48.51 ± 14.58	42.04 ± 11.63	0.000

25(OH)D (ng/mL)	Han	19.86 ± 7.18	19.18 ± 8.88	0.017
	Uyghur	16.04 ± 6.01^a^	11.67 ± 7.28^a^	0.000

TSH (IU/mL)	Han	2.18 (1.51–3.20)	2.76 (1.83–4.16)	0.000
	Uyghur	1.89 (1.33–2.82)^a^	2.32 (1.47–3.97)^a^	0.007

TPOAb (IU/mL)	Han	24.21 (19.75–30.42)	27.54 (22.96–36.97)	0.000
	Uyghur	25 (19.57–33.14)^a^	28.28 (22.15–40.89)^a^	0.000

TgAb (IU/mL)	Han	27.30 (24.50–31.48)	30.24 (26.11–70.58)	0.000
	Uyghur	28.57 (24.48–32.65)^a^	32.48 (27.43–103.4)^a^	0.000

^a^Significantly different from Uyghurs (*P* ≤ 0.001).

TSH: thyroid-stimulating hormone; 25(OH)D: serum 25-hydroxyvitamin D; TPOAb: anti-thyroid peroxidase antibody; TgAb: anti-thyroid-globulin antibody.

**Table 2:** Comparison of clinical and laboratory characteristics based on the positivity of serum antibodies.

	TPOAb(+)	TgAb(+)	TPOAb(+)TgAb(+)
Male/female	64/176	15/91	28/181
Han (%)	117 (48.8%)	48 (45.3%)^a^	120 (57.4%)
Uyghur (%)	123 (51.2%)	58 (54.7%)	89 (42.6%)
Age	47.0 ± 14.27	47.5 ± 13.39	46.06 ± 13.06
TSH (IU/mL)	2.38 (1.46–3.81)	2.87 (1.60–4.14)	3.63 (2.18–6.43)^b^
25(OH)D (ng/mL)	15.44 (10.9–21.97)	13.61 (10.05–18.47)^b^	15.03 (11.62–20.12)

^a^Significantly different from Uyghurs (*P* < 0.05); ^b^significantly different from the other two groups (*P* < 0.01).

TSH: thyroid-stimulating hormone; 25(OH)D: serum 25-hydroxyvitamin D; TPOAb: anti-thyroid peroxidase antibody; TgAb: anti-thyroid-globulin antibody.

**Table 3:** Linear regression analysis with serum TgAb as a dependent variable.

	Male		Female	
	*β*	*P* value	*β*	*P* value
Age	−0.055	0.974	0.014	0.907
Ethnicity	−0.006	0.995	0.003	0.739
25(OH)D	−0.036	0.987	−0.121	0.014
TSH	0.003	0.985	0.072	0.009
TPOAb	0.740	0.000	0.767	0.000

**Table 4:** Linear regression analysis with serum TPOAb as a dependent variable.

	Male		Female	
	*β*	*P* value	*β*	*P* value
Age	0.002	0.000	−0.002	0.011
Ethnicity	0.063	0.912	0.048	0.724
25(OH)D	0.005	0.002	0.006	0.000
TSH	0.017	0.000	0.013	0.000
TgAb	0.548	0.000	0.507	0.000

**Table 5:** Determinants of positive serum thyroglobulin antibody.

	TgAb	
	Adjusted OR (95% CI)	*P* value
Age	0.999 (0.990–1.009)	0.855
Gender	3.157 (2.230–4.469)	0.000
Ethnicity	1.335 (1.002–1.778)	0.048
25(OH)D	1.156 (1.004–1.331)	0.043
TSH	1.380 (1.192–1.597)	0.000
